RETRACTED

# MiR-543 Inhibits the Migration and Epithelial-To-Mesenchymal Transition of TGF-β-Treated Endometrial Stromal Cells via the MAPK and Wnt/β-Catenin Signaling Pathways

**DOI:** 10.3389/pore.2021.1609761

**Published:** 2021-04-29

**Authors:** Linlin Wang, Dan Liu, Jun Wei, Liwei Yuan, Shiyun Zhao, Yani Huang, Jingwen Ma, Zhijuan Yang

**Affiliations:** ^1^ College of Clinical Medicine, Ningxia Medical University, Yinchuan, China; ^2^ Medical Experimental Center, General Hospital of Ningxia Medical University, Yinchuan, China; ^3^ Department of Gynecology, General Hospital of Ningxia Medical University, Yinchuan, China; ^4^ Key Laboratory of Ministry of Education for Fertility Preservation and Maintenance, Ningxia Medical University, Yinchuan, China

**Keywords:** molecular biology, miRNA-543, MAPK1, wnt/β-catenin, endometrial stromal cell

## Abstract

Intrauterine adhesion (IUA) is one of the most prevalent reproductive system diseases in females. MicroRNAs (miRNAs) are reported to be master regulators in a variety of diseases, including IUA, but the role of microRNA-543 (miR-543) in IUA remains to be elucidated. In this study, we observed that miR-543 was downregulated in transforming growth factor-beta (TGF-β)-treated endometrial stromal cells (ESCs). Functionally, we observed that miR-543 suppressed the migration, epithelial-to-mesenchymal transition (EMT), and inhibited expression of extracellular matrix (ECM) proteins in TGF-β-treated ESCs. Mechanistically, MAPK1 is targeted by miR-543 after prediction and screening. A luciferase reporter assay demonstrated that miR-543 complementarily binds with the 3′ untranslated region of mitogen-activated protein kinase 1 (MAPK1), and western blot analysis indicated that miR-543 negatively regulates MAPK1 protein levels. In addition, results from rescue assays showed that miR-543 inhibits the migration and EMT of TGF-β-treated ESCs by targeting MAPK1. In addition, we observed that miR-543 inactivates the Wnt/β-catenin signaling pathway through inhibiting the phosphorylation of MAPK1 and β-catenin. Finally, we confirmed that miR-543 represses migration, EMT and inhibits levels of ECM proteins in TGF-β-treated ESCs by targeting the Wnt/β-catenin signaling pathway. Our results demonstrated that miR-543 suppresses migration and EMT of TGF-β-treated ESCs by targeting the MAPK and Wnt/β-catenin pathways.

## Introduction

Intrauterine adhesion (IUA), also known as Asherman syndrome, is one of the most common endometrial lesion diseases [1]. Recently, due to increased endometrial injury and endometrial infection, the incidence of IUA has increased [2]. At the present, standard therapies for IUA, such as transcervical resection of adhesions, have been widely applied to cure patients with IUA, but the recurrence rate after treatment remains high [1, 3]. Specifically, severe IUA is closely related to secondary infertility and miscarriage [4–6]. Hence, improved understanding of the pathology of IUA is needed, and identifying potential molecular targets for IUA treatment is exigent.

RETRACTED

Stromal cells are one of the main cell populations in the endometrium, and they are crucial mediators of endometrial function [7, 8]. Therefore, we focused on endometrial stromal cells (ESCs) in this study. Endometrial fibrosis and excessive extracellular matrix (ECM) deposition are the most important pathological characteristics of IUA [9, 10]. Furthermore, numerous studies have indicated that transforming growth factor (TGF)-β is a cytokine that participates in regulating diverse biological functions, including cell proliferation, apoptosis, and differentiation [11, 12]. Importantly, previous studies have reported that TGF-β can induce endometrial fibrosis [13, 14] and TGF-β treated ESC can serve as the *in vitro* model of IUA [15, 16].

MicroRNAs (miRNAs) are indicated to play pivotal roles in a variety of diseases, including Alzheimer’s disease [17], glaucoma [18] and diabetes [19]. Importantly, the crucial roles of a great number of miRNAs in ESCs have been revealed. For instance, miR-205-5p was observed to inhibit endometriosis progression via ANGPT2 in ESCs [20]. MiR-26a facilitated apoptosis of ESCs by direct regulation of PTEN and indirect regulation of the PI3K/AKT signaling [21]. It was reported that miR-320a boosts the migration of human ESCs [22]. MicroRNA-543 (miR-543) was demonstrated to exert a crucial effect on several tumors, such as hepatocellular carcinoma [23] and osteosarcoma [24]. Endogenous miR-543 expression is decreased in malignant endometrium tissues compared to that in normal endometrium tissues, and forced expression of miR-543 inhibits monolayer proliferation, anchorage-independent growth, migration and invasion of endometrial cancer cells [25]. Endometriosis is an important cause of intrauterine adhesion. MiR-543 was significantly downregulated in the eutopic endometrium in patients with endometriosis [26]. Previously, miR-543 was identified to be downregulated in IUA tissues [27]. However, whether miR-543 plays a role in ESCs has not been explored.

In the present study, we focused on the role of miR-543 in TGF-β-treated ESCs. We first determined expression of miR-543 in TGF-β-treated ESCs, followed by the biological functions of miR-543 in TGF-β-treated ESCs. Subsequently, we investigated the molecular regulatory mechanism of miR-543 in TGF-β-treated ESCs. In conclusion, our results suggested that miR-543 inhibits migration and EMT of TGF-β-treated ESCs through the MAPK and Wnt/β-catenin signaling pathways.

RETRACTED

## Materials and Methods

### Cell Culture and Treatment

THESCs (telomerase immortalized cell line; catalogue number: CRL-4003) [28] were obtained from the American Type Culture Collection (ATCC; United States). All cells were cultured in Dulbecco’s modified Eagle’s medium (DMEM; United States) with 10% fetal bovine serum (FBS; Invitrogen, United States), 100 U/ml penicillin (Sigma-Aldrich, United States) and 100 μg/ml streptomycin (Sigma-Aldrich, United States) and maintained in the humidified incubator containing 5% CO_2_ at 37°C. For cell treatment, ESCs were seeded into 6-well plates (2 × 10^5^ cells per well) and treated with different concentrations of TGF-β1 (0, 5, 10, or 15 ng/ml; Boehringer). After 48 h, cells were harvested for cell viability assay. For some groups, cells were cotreated with MAPK inhibitor SB 203580 (S8307; Sigma-Aldrich) dissolved in DMSO at concentration of 20 umol/L, TGF-beta1 specific inhibitor disitertide (M9083; AbMole) dissolved in DMSO at concentration of 5 mmol/L, as well as activator of Wnt/β-catenin signaling LiCl (L9650; Sigma-Aldrich) dissolved in DMSO at concentration of 10 mmol/L and KCl (P3911; Sigma-Aldrich) dissolved in DMSO at concentration of 10 mmol/L for 48 h.

### Transfection

MiR-543 mimics were used for miR-543 overexpression with NC mimics as the negative control. The pcDNA3.1 vector carrying full length mitogen-activated protein kinase 1 (MAPK1) was designed to overexpress MAPK1 with an empty pcDNA3.1 vector as a negative control. All plasmids were purchased from RiboBio Co., Ltd. (Guangzhou, China). Transfections of miR-543 mimics (50 μM) and pcDNA3.1-MAPK1 (2 μg) were performed using Lipofectamine 2000 (Invitrogen; Thermo Fisher Scientific, Inc.) at 37°C for 24 h. After transfection for 24 h, cells were treated with 10 ng/ml TGF-β1 for 48 h.

### RNA Extraction and Reverse Transcription Quantitative Polymerase Chain Reaction

After washing in PBS three times and centrifugation at 800 x g for 20 min at 4°C, total RNA was extracted from cells using TRIzol reagent (Invitrogen, United States) following the manufacturer’s instructions. Total RNA (2 μg) was reverse transcribed into cDNA using a High-Capacity cDNA Reverse Transcription Kit (Applied Biosystems, United States) at 42°C for 60 min and 82°C for 10 s. Quantitative PCR was conducted using Power SYBR Green RT-PCR reagents (Applied Biosystems). All reactions were performed on an Applied Biosystems 7000 Sequence Detection System (Applied Biosystems). The thermocycling conditions were as follows: denaturation at 94°C for 5 min, amplification for 40 cycles at 94°C for 30 s, annealing at 60°C for 30 s and extension at 72°C for 1 min. The detection results for mRNAs were normalized to GAPDH. U6 served as the endogenous control for miRNA. Expression fold changes were calculated adopting the 2^−ΔΔCt^ method [29]. Primer sequences are listed in Supplementary Table S1. Each biological sample was run in triplicate and experiments were independently repeated three times.

RETRACTED

### Western Blot Analysis

Transfected cells were lyzed in RIPA buffer (Thermo, United States) and incubated at 4°C for 15 min. The lysate was centrifuged, and protein concentration was detected using a BCA Protein Assay Kit (Thermo, United States). Separation of cytoplasmic and nuclear proteins for western blot is performed using a Subcellular Protein Fractionation Kit for Cultured Cells (Thermo Scientific) according to the manufacturer’s instructions. Protein samples (30 μg/lane) were isolated on 10% sodium dodecyl sulfate polyacrylamide gel electrophoresis and transferred onto polyvinylidene fluoride membranes (Thermo, United States. Then, membranes were blocked using 5% skim milk for 1 h and incubated with primary antibodies at 4°C overnight. Primary antibodies were used as follows: collagen I (ab34710, Abcam), collagen III (ab7778, Abcam), fibronectin (ab2413, Abcam), α-SMA (ab32575, Abcam), E-cadherin (ab1416, Abcam), Vimentin (ab8069, Abcam), N-cadherin (ab18203, Abcam), MAPK1 (ab184699, Abcam), p-MAPK1 (ab131438, Abcam), β-catenin (ab32572, Abcam), p-β-catenin (ab53050, Abcam), prolactin (ab183967, Abcam), desmin (ab32362, Abcam), GAPDH (ab8245, Abcam), tubulin (ab6160, Abcam), and laminA/C (ab108595, Abcam). Subsequently, membranes were incubated with goat anti-mouse (ab205719, Abcam) or goat anti-rabbit (ab6721, Abcam) secondary antibodies (conjugation: horse radish peroxidase; Isotype: IgG) at room temperature for 2 h. Finally, an enhanced chemiluminescence kit (GE Healthcare, Chicago, IL, United States) was adopted to observe the signals. Each biological sample was run in triplicate and experiments were independently repeated three times.

### Luciferase Reporter Assay

Wild type or mutant sequences of MAPK1 3′ UTR were cloned into pmirGLO reporters (Promega, United States). MAPK1 3′ UTR-Wt or MAPK1 3′ UTR-Mut vectors were cotransfected with miR-543 mimics or NC mimics, respectively, into ESCs. Lipofectamine 2000 (Invitrogen) was used for the transfections. Forty-eight hours later, luciferase reporter assays were used to examine the relative luciferase activities. Each biological sample was run in triplicate and experiments were independently repeated three times.

### Immunofluorescence Staining

Transfected ESCs were cultured on the surface of 8 mm × 8 mm slide in 24-well plates and fixed in ethanol for 15 min. Then, slides were washed in distilled H_2_O and PBS three times. Next, slides were blocked in normal serum for 30 min at room temperature. Slides were then incubated with anti-β-catenin antibody (ab32572, Abcam) overnight at 4°C. Subsequently, goat polyclonal alexa Fluor® 488 conjugated secondary antibodies (ab150077, Abcam) were added, and cells were incubated for another 2 h at room temperature. Finally, the slides were washed in PBS and observed under a confocal microscope (FluoView FV500; Olympus). Each biological sample was run in triplicate and experiments were independently repeated three times.

RETRACTED

### TOP-Flash Assay

When the Wnt/β-catenin pathway is activated, β-catenin is translocated to the nucleus, where in complexes with members of the TCF/LEF family of transcription regulators, activates transcription of TCF-responsive genes. TOP-Flash is a TCF-reporter plasmid, along with FOP-Flash enables quantitation of the Wnt/β-catenin signaling in cells transfected with these constructs. TOP/FOP-Flash (Genechem) was cotransfected into cells with NC mimics, miR-543 mimics, miR-543 + pcDNA3.1, miR-543 + MAPK1. The pRL-SV40 vector (Promega) that encodes renilla luciferase gene was used to standardize the transfection efficiency. Luciferase assay was conducted with the Dual Luciferase Assay System kit 36 h after transfection. Relative luciferase activity is reported as fold induction (TOP/FOP) after normalization for transfection efficiency. Each biological sample was run in triplicate and experiments were independently repeated three times.

### MTT Assay

The viability of ESCs was assessed using the MTT assay. ESCs were seeded into 96‐well plates with 5 × 10^3^ cells/well. Each well was supplemented with 100 μl fresh DMEM and 0.5 mg ml^−1^ MTT at 48 h, and the incubation continued for 4 h at 37°C. Then, the medium was replaced with 100 μl DMSO, and absorbance was measured at 490 nm to calculate the OD value. Cell viability (%) = (OD[Experiment]-OD[blank])/(OD[control]-OD[blank]) × 100%. OD[blank] refers to the OD of plate with medium and MTT solution but without cells. OD[control] refers to the OD of plate in normal condition. Each biological sample was run in triplicate and experiments were independently repeated three times.

### Wound Healing Assay

Wound healing assay was performed to detect ESC migration. Transfected cells were plated into 6-well plates at a density of 1 × 10^5^ cells per well. Then, a sterile plastic micropipette tip was applied to scratch the center of the plate. Cell movement was recorded using Image-Pro Plus 6.0 software. Each biological sample was run in triplicate and experiments were independently repeated three times.

RETRACTED

### Transwell Assay

Transwell assays were performed to evaluate the migratory capability of ESCs. After TGF-β1 treatment for 2 days, ESCs were digested with trypsin and washed with PBS. Serum-free medium cultured ESCs in each group were digested with trypsin and plated in the upper chamber with 2 × 10^4^ cells/100 μl and incubated in serum-free medium. The lower chambers received 600 μl DMEM containing 10% FBS. After 24 h, cells were fixed in 4% paraformaldehyde, stained with 0.1% crystal violet for 10 min. Then, cells were washed in PBS three times. Finally, five fields were randomly selected for analysis from each sample. Each biological sample was run in triplicate and experiments were independently repeated three times.

### Statistical Analysis

All experiments were repeated three times. Statistical analysis was performed with SPSS 13.0, and graphs were constructed in GraphPad Prism 5 (La Jolla, CA, United States). Data are shown as the mean ± standard deviation. Significant differences between groups were assessed by Student’s t-test and one-way analysis of variance followed by Tukey’s *post hoc* analysis and Dunnett’s *post hoc* tests. *p* < 0.05 was considered to be significant.

## Results

### MiR-543 is Downregulated in TGF-β-Treated ESCs, and miR-543 Overexpression Inhibits ECM Protein Levels, Suppresses Migration and EMT of TGF-β- Treated ESCs

As shown in Figure 1A, ESCs were treated with different concentrations of TGF-β (0 ng/ml, 5 ng/ml, 10 ng/ml, or 15 ng/ml). Cells in the “Control” group lack both TGF-β treatment and transfections. MTT assay showed that treatment with increasing concentrations of TGF-β induced a gradual decrease in ESC viability. We observed that miR-543 was downregulated in TGF-β-treated ESCs compared to the control group (Figure 1B). Next, we found that miR-543 was distinctly overexpressed by transfecting miR-543 mimics into TGF-β-treated ESCs (Figure 1C). Overexpression of miR-543 significantly promoted cell viability (Figure 1D). Subsequently, western blot analysis revealed that TGF-β induced increase of ECM proteins including collagen I, collagen III, α-SMA and fibronectin, while overexpression of miR-543 significantly decreased levels of ECM proteins (Figure 1E). Moreover, the results of wound healing (Figures 1F,G) and Transwell assays revealed that TGF-β treatment caused the promoted migration and invasion of ESCs, while miR-543 overexpression reduced the migratory capability of TGF-β-treated ESCs (Figure 1H). Furthermore, we found that TGF-β treatment promoted expression of mesenchymal cell markers N-cadherin and Vimentin and reduced expression of epithelial cell marker E-cadherin; overexpression of miR-543 decreased the levels of N-cadherin and Vimentin, while increased levels of E-cadherin, as revealed in western blot analysis (Figure 1I) and immunofluorescence staining assay (Figures 1J,K). TGF-β treatment or miR-543 overexpression had no effects on protein levels of prolactin and desmin in ESCs (Supplementary Figure S1).

RETRACTED

**FIGURE 1:** MiR-543 overexpression exerts an inhibitory effect on ECM protein levels, migration and EMT of TGF-β-treated ESCs. **(A)** The effect of TGF-β1 on the viability of ESCs after treatment of different concentrations of TGF-β1 for 48 h was detected by MTT. **(B)** Expression of miR-543 in ESCs after treatment of TGF-β1 for 48 h was determined by RT-qPCR. **(C)** The efficiency of miR-543 overexpression was detected after 24 h of transfection followed by 48 h of TGF-β1 treatment. **(D)** MTT assay revealed the influence of miR-543 on cell viability of ESCs after 24 h of transfection followed by 48 h of TGF-β1 treatment. **(E)** Levels of proteins associated with fibrosis (collagen I, collagen III, α-SMA and fibronectin) in ESCs after 24 h of transfection followed by 48 h of TGF-β1 treatment were evaluated by western blot analysis. **(F–H)** Wound healing and transwell assays were performed to assess the migration of ESCs after 24 h of transfection followed by 48 h of TGF-β1 treatment. **(I)** Levels of mesenchymal cell markers (N-cadherin and Vimentin) and an epithelial cell marker (E-cadherin) in ESCs after 24 h of transfection followed by 48 h of TGF-β1 treatment were examined through western blot analysis. **(J–K)** Immunofluorescence staining assay revealed expression of E-cadherin, N-cadherin, and Vimentin in ESCs after 24 h of transfection followed by 48 h of TGF-β1 treatment. *p < 0.05, **p < 0.01, ***p < 0.001.

### MAPK1 is Targeted By miR-543 in TGF-β-Treated ESCs

Using the miRDB website (http://mirdb.org), we identified 1208 mRNAs sharing a binding site with miR-543. The top 10 mRNAs were selected for RT-qPCR analysis, and results revealed that expression of MAPK1 was markedly reduced in response to miR-543 overexpression (Figure 2A). Next, RT-qPCR analysis demonstrated that MAPK1 mRNA was highly expressed in TGF-β-treated ESCs compared to control ESCs (Figure 2B). Similarly, we observed that protein levels of MAPK1 were upregulated induced by TGF-β in ESCs compared to the control group (Figure 2C). To verify binding between MAPK1 and miR-543, a luciferase reporter assay was performed. The predicted binding site between MAPK1 and miR-543 is shown in Figure 2D. According to the results of luciferase reporter assay, luciferase activity in the MAPK1 Wt + miR-543 mimics group was lower than in the MAPK1 Wt + NC mimics group, while no significant difference was observed between MAPK1 Mut + miR-543 mimics and MAPK1 Mut + NC mimics groups (Figure 2D). Furthermore, we observed decreased MAPK1 protein in response to augmented miR-543 (Figure 2E).

RETRACTED

**FIGURE 2:** MiR-543 targets MAPK1 in TGF-β-treated ESCs. **(A)** 1208 target mRNAs for miR-543 were predicted by http://mirdb.org. The effect of miR-543 overexpression on the top 10 mRNAs in ESCs after 24 h of transfection was analyzed by RT-qPCR. **(B)** Levels of MAPK1 mRNA and **(C)** protein in ESCs treated with TGF-β for 48 h were assessed. **(D)** The binding site between miR-543 and MAPK1. The binding capacity between miR-543 and MAPK1 in ESCs after 48 h of transfection was assessed using a luciferase reporter assay. **(E)** The effect of miR-543 overexpression on levels of MAPK1 protein in ESCs after 24 h of transfection followed by 48 h of TGF-β1 treatment. *p < 0.05, **p < 0.01.

### MiR-543 Regulates ECM Protein Levels, Migration, and EMT of TGF-β-Treated ESCs by Targeting MAPK1

Subsequently, we further investigated the potential regulatory mechanism of miR-543 in TGF-β-treated ESCs. First, levels of MAPK1 mRNA and protein were observed to be markedly increased after the transfection of pcDNA3.1/MAPK1 into TGF-β-treated ESCs (Figure 3A). MTT assay results demonstrated that increased MAPK1 offset the promotion of cell viability arising from miR-543 overexpression (Figure 3B). The decreased ECM protein levels induced by miR-543 mimics was restored by MAPK1 overexpression in TGF-β-treated ESCs (Figure 3C). In addition, overexpressed MAPK1 rescued the inhibitory effect of miR-543 overexpression on the migration of TGF-β-treated ESCs (Figures 3D,E). Furthermore, miR-543 mimics-induced decreases in levels of mesenchymal cell markers (N-cadherin and Vimentin) and increased levels of epithelial cell marker (E-cadherin) were rescued by MAPK1 overexpression (Figure 3F).

**FIGURE 3:** MiR-543 represses ECM protein levels, migration, and EMT of TGF-β-treated ESCs through regulation of MAPK1. **(A)** The overexpression efficiency of MAPK1 in ESCs after 24 h of transfection followed by 48 h of TGF-β1 treatment was detected. **(B)** Cell viability of ESCs after 24 h of transfection followed by 48 h of TGF-β1 treatment in NC mimics, miR-543 mimics, miR-543 mimics + vector, and miR-543 mimics + MAPK1 groups was assessed by MTT assay. **(C)** Western blot analysis showing protein levels of collagen I, collagen III, α-SMA and fibronectin of ESCs after 24 h of transfection followed by 48 h of TGF-β1 treatment in the four groups. **(D, E)** The migratory capability of ESCs after 24 h of transfection followed by 48 h of TGF-β1 treatment in the 4 groups. **(F)** Levels of mesenchymal cell markers (N-cadherin and Vimentin) and an epithelial cell marker (E-cadherin) of ESCs after 24 h of transfection followed by 48 h of TGF-β1 treatment were examined. *p < 0.05, **p < 0.01, ***p < 0.001.

RETRACTED

### MiR-543 Inactivated the Wnt/β-Catenin Signaling Pathway by Targeting MAPK1

Through western blot analysis, we observed that miR-543 overexpression reduced the protein levels of Wnt, MAPK1, phosphorylated MAPK1 and β-catenin, which was rescued by MAPK1 overexpression (Figure 4A). Overexpression of miR-543 suppressed protein levels of N-cadherin and Vimentin, while increasing protein levels of E-cadherin. Treatment with SB 203580 further suppressed protein levels of N-cadherin and Vimentin, as well as increased protein levels of E-cadherin (Figure 4B). Protein levels of phosphorylated Smad2/3 were activated by TGF-β1 and were reduced by miR-543, while Smad7 protein exhibited the opposite trend. Treatment with disitertide (an inhibitor of TGF-β) significantly reduced protein levels of phosphorylated Smad2/3 and increased levels of Smad7 (Figure 4C). Furthermore, according to the results of immunofluorescence staining, we observed that miR-543 overexpression inhibited nuclear translocation of β-catenin, while MAPK1 overexpression led to nuclear translocation of β-catenin (Figure 4D). Meanwhile, nuclear accumulation of β-catenin was inhibited by miR-543 overexpression and was facilitated by MAPK1 overexpression (Figure 4E). Moreover, overexpression of miR-543 inhibited TOP/FOP reporter activity, which was rescued by overexpression of MAPK1 (Figure 4F).

**FIGURE 4:** MAPK1 overexpression offsets miR-543 overexpression-induced inactivation of the Wnt/β-catenin signaling pathway. **(A)** Levels of Wnt/β-catenin signaling pathway-associated proteins, Wnt, p-MAPK1, MAPK1, p-β-catenin, and β-catenin in ESCs after transfection of NC mimics, miR-543 mimics, miR-543 mimics + vector and miR-543 mimics + MAPK1 for 24 h followed by 48 h of TGF-β1 treatment. **(B)** Levels of E-cadherin, N-cadherin and Vimentin in NC mimics, miR-543 mimics, miR-543 mimics + SB 203580 groups in ESCs after 24 h of transfection followed by 48 h of TGF-β1 and SB 203580 treatment. **(C)** Levels of p-Smad2/3, Smad7 in ESCs after 24 h of transfection followed by 48 h of TGF-β1 and disitertide treatment. **(D)** Immunofluorescence images of ESCs transfected with NC mimics, miR-543 mimics, miR-543 mimics + vector and miR-543 mimics + MAPK1 for 24 h followed by 48 h of TGF-β1 treatment. **(E)** Localization of β-catenin in ESCs was detected after transfection with NC mimics, miR-543 mimics, miR-543 mimics + vector and miR-543 mimics + MAPK1 for 24 h followed by 48 h of TGF-β1 treatment. **(F)** Activity of the TOP/FOP reporter plasmid in ESCs after 36 h of transfection followed by 48 h of TGF-β1 treatment was detected by the TOP/FOP flash assay. *p < 0.05, **p < 0.01, ***p < 0.001.

RETRACTED

### MiR-543 Regulates Migration and EMT of TGF-β-Treated ESCs Through the Wnt/β-Catenin Signaling Pathway

To confirm whether activation of the Wnt/β-catenin signaling pathway can rescue the repressive effect of miR-543 overexpression on migration and EMT of TGF-β-treated ESCs, TGF-β-treated ESCs were transfected with miR-543 mimics or NC mimics and treated with LiCl, or KCI (negative control for LiCl). Results from the TOP/FOP flash assay suggested that introduction of LiCl offset the inhibition of TOP/FOP reporter activity arising from miR-543 overexpression (Figure 5A). In addition, miR-543 mimics-induced inhibition of cell viability was abolished by LiCl (Figure 5B). LiCl treatment rescued the repressive effect of miR-543 overexpression on ECM protein levels, including collagen I, collagen III, α-SMA and fibronectin (Figure 5C). Additionally, LiCl treatment rescued the inhibitory effect of miR-543 overexpression on the migration of TGF-β-treated ESCs (Figures 5D,E). Moreover, miR-543 overexpression-induced decreases in levels of mesenchymal cell markers (N-cadherin and Vimentin) and increases in levels of the epithelial cell marker (E-cadherin) were rescued by LiCl treatment (Figure 5F).

**FIGURE 5:** MiR-543 suppresses migration and EMT of TGF-β- treated ESCs through the Wnt/β-catenin signaling pathway. **(A)** Activity of the TOP/FOP reporter plasmid in NC mimics, miR-543 mimics, miR-543 mimics + KCI and miR-543 mimics + LiCl groups of ESCs in ESCs after 36 h of transfection followed by 48 h of TGF-β1 and LiCl (or KCl) treatment. **(B)** Cell viability of the four groups of ESCs after 24 h of transfection followed by 48 h of TGF-β1 and LiCl (or KCl) treatment. **(C)** Protein levels of collagen I, collagen III, α-SMA and fibronectin in the four groups of ESCs after 24 h of transfection followed by 48 h of TGF-β1 and LiCl (or KCl) treatment. **(D, E)** Migratory capability of TGF-β-treated ESCs in the four groups of ESCs after 24 h of transfection followed by 48 h of TGF-β1 and LiCl (or KCl) treatment. **(F)** Levels of EMT associated proteins in ESCs of the four groups of ESCs after 24 h of transfection followed by 48 h of TGF-β1 and LiCl (or KCl) treatment. **p < 0.01, ***p < 0.001.

## Discussion

Over the last several decades, IUA incidence has rapidly increased, although there are many treatments for this disease [5]. Currently, patients with IUA are confronted with the huge risk of secondary infertility and recurrent miscarriage [2]. Therefore, an improved understanding of IUA is indispensable.

RETRACTED

Previous studies have revealed that miRNAs play a significant role in the regulation of ESCs [20–22]. Recently, miR-543 has attracted great attention, and the role of miR-543 has been investigated in a variety of diseases [30]. For instance, it was reported that miR-543 enhances the migratory and invasive capabilities of esophageal cancer cells [31]. MiR-543 was also found to promote cell proliferation and EMT of prostate cancer through the regulation of RKIP [32]. Furthermore, miR-543 regulates the epigenetic landscape of myelofibrosis via TET1 and TET2 [33]. Importantly, miR-543 was demonstrated to be downregulated in IUA tissues [27]. In the current study, our results revealed that miR-543 was downregulated in TGF-β-treated ESCs. We also observed that miR-543 overexpression inhibits fibrotic changes, migration and EMT of TGF-β-treated ESCs.

MAPK1 is a widely studied gene that encodes a member of the MAP kinase family. MAP kinases, also known as extracellular signal-regulated kinases, participate in a wide variety of cellular processes such as proliferation, differentiation, transcription regulation and development [34, 35]. Specifically, MAPK1 was found to be involved in the regulation of IUA [36, 37]. In this study, we determined that MAPK1 is a downstream target of miR-543. MiR-543 repressed migration, EMT and fibrotic changes of TGF-β-treated ESCs through the regulation of MAPK1. In other words, miR-543 exerted a significant effect on TGF-β-treated ESCs via MAPK pathway. MiR-543 has been reported to target ERK2 and suppress the MAPK pathway [38]. Furthermore, previous studies have verified that MAPK1 facilitates the phosphorylation of β-catenin [34]. Consistently, our data verified that MAPK1 promotes phosphorylation of β-catenin. The Wnt/β-catenin signaling pathway is a common pathway that participates in the regulation of various diseases [39]. Previous studies revealed that miR-543 suppresses the Wnt/β-catenin signaling pathway in renal cell carcinoma [40] and in bladder cancer [41] by targeting DKK-1. Importantly, the Wnt/β-catenin signaling was found to be involved in regulating the phenotype of ESCs [42–44]. In the current study, we discovered that MAPK1 overexpression offset the inhibitory effect of miR-543 overexpression on protein levels of MAPK1 and β-catenin. In addition, we verified that miR-543 regulates migration, EMT and fibrotic changes of TGF-β-treated ESCs by directly targeting MAPK1 and the Wnt/β-catenin signaling pathway.

RETRACTED

In conclusion, our study aimed to reveal the biological role and regulatory mechanism of miR-543 in TGF-β-treated ESCs. Our results revealed that miR-543 inhibits ECM protein levels, suppresses migration and EMT of TGF-β-treated ESCs via inhibition on the MAPK and the Wnt/β-catenin signaling pathways by targeting MAPK1. These findings highlight the regulatory role of miR-543 in TGF-β-treated ESCs, which may shed light on the possible pathophysiological mechanisms of IUA. Evidence from *in vivo* experiments should be added in future studies.

## Data Availability

The original contributions presented in the study are included in the article/Supplementary Material, further inquiries can be directed to the corresponding authors.

## References

[1] HealyMWSchexnayderBConnellMTTerryNDeCherneyAHCsokmayJM. Intrauterine Adhesion Prevention after Hysteroscopy: a Systematic Review and Meta-Analysis. Am J Obstet Gynecol (2016) 215(3):267–75. 10.1016/j.ajog.2016.05.001 27173082

[2] TamWHLauWCCheungLPYuenPMChungTK-H. Intrauterine adhesions after conservative and surgical management of spontaneous abortion. The J Am Assoc Gynecol Laparoscopists (2002) 9(2):182–5. 10.1016/s1074-3804(05)60129-6 11960045

[3] LudwinAMartinsWPLudwinI. Ultrasound-guided repeat intrauterine balloon dilatation for prevention of adhesions. Ultrasound Obstet Gynecol (2019) 54:566–8. 10.1002/uog.20223 30677188

[4] LaganàASGarzonSFranchiMCasarinJGulloGGhezziF. Translational animal models for endometriosis research: a long and windy road. Ann Transl Med (2018) 6(22):431. 10.21037/atm.2018.08.24 30596061PMC6281523

[5] FeiZBinZXinXFeiHYuechongC. Meta-analysis on the use of hyaluronic acid gel to prevent recurrence of intrauterine adhesion after hysteroscopic adhesiolysis. Taiwanese J Obstet Gynecol (2019) 58(6):731–6. 10.1016/j.tjog.2019.09.002 31759520

[6] YuDWongY-MCheongYXiaELiT-C. Asherman syndrome-one century later. Fertil sterility (2008) 89(4):759–79. 10.1016/j.fertnstert.2008.02.096 18406834

[7] MaslarIARiddickDH. Prolactin production by human endometrium during the normal menstrual cycle. Am J Obstet Gynecol (1979) 135(6):751–4. 10.1016/0002-9378(79)90386-7 495675

[8] IrwinJCKirkDKingRJBQuigleyMMGwatkinRBL. Hormonal regulation of human endometrial stromal cells in culture: an in vitro model for decidualization. Fertil sterility (1989) 52(5):761–8. 10.1016/s0015-0282(16)61028-2 2806617

[9] ZhuH-YGeT-XPanY-BZhangS-Y. Advanced role of hippo signaling in endometrial fibrosis. Chin Med J (2017) 130(22):2732–7. 10.4103/0366-6999.218013 29133764PMC5695061

[10] GuoLPChenLMChenFJiangNHSuiL. Smad signaling coincides with epithelial-mesenchymal transition in a rat model of intrauterine adhesion. Am J Transl Res (2019) 11(8):4726–37. 31497194PMC6731410

RETRACTED

[11] SpornMBRobertsAB. TGF-beta: problems and prospects. Cell Regul (1990) 1(12):875–82. 10.1091/mbc.1.12.875 2100192PMC362858

[12] KamatoDBurchMLPivaTJRezaeiHBRostamMAXuS. Transforming growth factor-β signalling: Role and consequences of Smad linker region phosphorylation. Cell Signal (2013) 25(10):2017–24. 10.1016/j.cellsig.2013.06.001 23770288

[13] BaiXLiuJYuanWLiuYLiWCaoS. Therapeutic effect of human amniotic epithelial cells in rat models of intrauterine adhesions. Cel Transpl (2020) 29:096368972090849. 10.1177/0963689720908495 PMC744421432223314

[14] SongMCaoCZhouZYaoSJiangPWangH. HMGA2-induced epithelial-mesenchymal transition is reversed by let-7d in intrauterine adhesions. Mol Hum Reprod (2021) 27(2). 10.1093/molehr/gaaa074 PMC786400333237328

[15] AiYChenMLiuJRenLYanXFengY. lncRNA TUG1 promotes endometrial fibrosis and inflammation by sponging miR-590-5p to regulate Fasl in intrauterine adhesions. Int immunopharmacol. (2020) 86:106703. 10.1016/j.intimp.2020.106703 32599321

[16] CaoJLiuDZhaoSYuanLHuangYMaJ. Estrogen attenuates TGF-β1-induced EMT in intrauterine adhesion by activating Wnt/β-catenin signaling pathway. Braz J Med Biol Res (2020) 53(8):e9794. 10.1590/1414-431x20209794 32638833PMC7346761

[17] CaoJHuangMGuoLZhuLHouJZhangL. MicroRNA-195 rescues ApoE4-induced cognitive deficits and lysosomal defects in Alzheimer's disease pathogenesis. Mol Psychiatry (2020). 10.1038/s41380-020-0824-3 PMC778568532632205

[18] DrewryMDChallaPKuchteyJGNavarroIHelwaIHuY. Differentially expressed microRNAs in the aqueous humor of patients with exfoliation glaucoma or primary open-angle glaucoma. Hum Mol Genet (2018) 27(7):1263–75. 10.1093/hmg/ddy040 29401312PMC6048986

[19] TorellaDIaconettiCTaralloRMarinoFGiuratoGVenezianoC. miRNA regulation of the hyperproliferative phenotype of vascular smooth muscle cells in diabetes. Diabetes (2018) 67(12):2554–68. 10.2337/db17-1434 30257973

[20] ZhouC-FLiuM-JWangWWuSHuangY-XChenG-B. miR-205-5p inhibits human endometriosis progression by targeting ANGPT2 in endometrial stromal cells. Stem Cel Res Ther (2019) 10(1):287. 10.1186/s13287-019-1388-5 PMC675739131547870

[21] ZhangLLiuXLiuJMaXZhouZSongY. miR-26a promoted endometrial epithelium cells (EECs) proliferation and induced stromal cells (ESCs) apoptosis via the PTEN -PI3K/AKT pathway in dairy goats. J Cel Physiol (2018) 233(6):4688–706. 10.1002/jcp.26252 29115668

[22] BerkhoutRPKeijserRReppingSLambalkCBAfinkGBMastenbroekS. High-quality human preimplantation embryos stimulate endometrial stromal cell migration via secretion of microRNA hsa-miR-320a. Hum Reprod (2020). 10.1093/humrep/deaa149 PMC739862332644109

RETRACTED

[23] YuLZhouLChengYSunLFanJLiangJ. MicroRNA-543 acts as an oncogene by targeting PAQR3 in hepatocellular carcinoma. Am J Cancer Res (2014) 4(6):897–906. 25520877PMC4266721

[24] WangL-HTsaiH-CChengY-CLinC-YHuangY-LTsaiC-H. CTGF promotes osteosarcoma angiogenesis by regulating miR-543/angiopoietin 2 signaling. Cancer Lett (2017) 391:28–37. 10.1016/j.canlet.2017.01.013 28108312

[25] BingLHongCLi-XinSWeiG. MicroRNA-543 suppresses endometrial cancer oncogenicity via targeting FAK and TWIST1 expression. Arch Gynecol Obstet (2014) 290(3):533–41. 10.1007/s00404-014-3219-3 24699721

[26] YangPWuZMaCPanNWangYYanL. Endometrial miR-543 is downregulated during the implantation window in women with endometriosis-related infertility. Reprod Sci (2019) 26(7):900–8. 10.1177/1933719118799199 30231774

[27] LiuXDuanHZhangH-HGanLXuQ. Integrated data set of microRNAs and mRNAs involved in severe intrauterine adhesion. Reprod Sci (2016) 23(10):1340–7. 10.1177/1933719116638177 27052751

[28] KrikunGMorGAlveroAGullerSSchatzFSapiE. A novel immortalized human endometrial stromal cell line with normal progestational response. Endocrinology (2004) 145(5):2291–6. 10.1210/en.2003-1606 14726435

[29] LivakKJSchmittgenTD. Analysis of relative gene expression data using real-time quantitative PCR and the 2−ΔΔCT method. Methods (2001) 25(4):402–8. 10.1006/meth.2001.1262 11846609

[30] ZhouCZhaoXDuanS. The role of miR‐543 in human cancerous and noncancerous diseases. J Cel Physiol (2020) 236:15. 10.1002/jcp.29860 32542683

[31] ZhaoHDiaoCWangXXieYLiuYGaoX. MiR-543 promotes migration, invasion and epithelial-mesenchymal transition of esophageal cancer cells by targeting phospholipase A2 group IVA. Cell Physiol Biochem (2018) 48(4):1595–604. 10.1159/000492281 30071514

[32] DuYLiuX-HZhuH-CWangLNingJ-ZXiaoC-C. MiR-543 promotes proliferation and epithelial-mesenchymal transition in prostate cancer *via* targeting RKIP. Cel Physiol Biochem (2017) 41(3):1135–46. 10.1159/000464120 28245474

[33] Fuentes-MatteiEBayraktarRManshouriTSilvaAMIvanCGuleiD. miR-543 regulates the epigenetic landscape of myelofibrosis by targeting TET1 and TET2. JCI insight (2020) 5(1). 10.1172/jci.insight.121781 PMC703082331941838

[34] ZhengYZhouCYuX-XWuCJiaH-LGaoX-M. Osteopontin promotes metastasis of intrahepatic cholangiocarcinoma through recruiting MAPK1 and mediating Ser675 phosphorylation of β-Catenin. Cell Death Dis (2018) 9(2):179. 10.1038/s41419-017-0226-x 29415992PMC5833342

[35] WangDPTangXZLiangQKZengXJYangJBXuJ. Overexpression of long noncoding RNA SLC26A4‐AS1 inhibits the epithelial-mesenchymal transition via the MAPK pathway in papillary thyroid carcinoma. J Cel Physiol (2020) 235(3):2403–13. 10.1002/jcp.29145 31556116

RETRACTED

[36] LiuSHuangXLiuYSongDXiaoY. Functional analysis of miRNAs combined with TGF-β1/Smad3 inhibitor in an intrauterine rat adhesion cell model. Mol Cel Biochem (2020) 470(1–2):15–28. 10.1007/s11010-020-03741-7 32447720

[37] LucchiNWMooreJM. LPS induces secretion of chemokines by human syncytiotrophoblast cells in a MAPK-dependent manner. J Reprod Immunol (2007) 73(1):20–7. 10.1016/j.jri.2006.05.005 16870263

[38] ChenPXuWLuoYZhangYHeYYangS. MicroRNA 543 suppresses breast cancer cell proliferation, blocks cell cycle and induces cell apoptosis via direct targeting of ERK/MAPK. Ott (2017) 10:1423–31. 10.2147/ott.S118366 PMC534806828331335

[39] HuangPYanRZhangXWangLKeXQuY. Activating Wnt/β-catenin signaling pathway for disease therapy: challenges and opportunities. Pharmacol Ther (2019) 196:79–90. 10.1016/j.pharmthera.2018.11.008 30468742

[40] ChenZ-YDuYWangLLiuX-HGuoJWengX-D. MiR-543 promotes cell proliferation and metastasis of renal cell carcinoma by targeting Dickkopf 1 through the Wnt/β-catenin signaling pathway. J Cancer (2018) 9(20):3660–8. 10.7150/jca.27124 30405834PMC6216004

[41] GaoRLChenXRLiYNYanXYSunJGHeQL. Upregulation of miR-543-3p promotes growth and stem cell-like phenotype in bladder cancer by activating the Wnt/β-catenin signaling pathway. Int J Clin Exp Pathol (2017) 10(9):9418–26. 31966814PMC6965893

[42] LvYZhangLMaJFeiXXuKLinJ. CTHRC1 overexpression promotes ectopic endometrial stromal cell proliferation, migration and invasion via activation of the Wnt/β-catenin pathway. Reprod Biomed Online (2020) 40(1):26–32. 10.1016/j.rbmo.2019.10.001 31787549

[43] YiTLiuMLiXLiuXDingYHeJ. Benzo(a)pyrene inhibits endometrial cell apoptosis in early pregnant mice via the WNT5A pathway. J Cel Physiol (2019) 234(7):11119–29. 10.1002/jcp.27762 30443902

[44] ZhouQYanGDingLLiuJYuXKongS. EHD1 impairs decidualization by regulating the Wnt4/β-catenin signaling pathway in recurrent implantation failure. EBioMedicine (2019) 50:343–54. 10.1016/j.ebiom.2019.10.018 31707150PMC6921214

